The article "Breast Tumor Detection and Classification in Mammogram Images Using Modified YOLOv5 Network" was retracted in 2023. Reasons: unreliable results or conclusions; concerns about the data; concerns about the peer review; concerns about the citations.

# Breast Tumor Detection and Classification in Mammogram Images Using Modified YOLOv5 Network

**DOI:** 10.1155/2022/1359019

**Published:** 2022-01-04

**Authors:** Aqsa Mohiyuddin, Asma Basharat, Usman Ghani, Veselý Peter, Sidra Abbas, Osama Bin Naeem, Muhammad Rizwan

**Affiliations:** ^1^Department of Computer Science, Kinnaird College for Women Lahore, Pakistan; ^2^University of Engineering and Technology Lahore, Pakistan; ^3^Information Systems Department, Faculty of Management, Comenius University in Bratislava, Odbojárov 10 82005 Bratislava 25, Slovakia; ^4^Department of Computer Science, COMSATS University, Sahiwal, Pakistan; ^5^University of Engineering and Technology Narowal, Pakistan

## Abstract

Breast cancer incidence has been rising steadily during the past few decades. It is the second leading cause of death in women. If it is diagnosed early, there is a good possibility of recovery. Mammography is proven to be an excellent screening technique for breast tumor diagnosis, but its detection and classification in mammograms remain a significant challenge. Previous studies' major limitation is an increase in false positive ratio (FPR) and false negative ratio (FNR), as well as a drop in Matthews correlation coefficient (MCC) value. A model that can lower FPR and FNR while increasing MCC value is required. To overcome prior research limitations, a modified network of YOLOv5 is used in this study to detect and classify breast tumors. Our research is conducted using publicly available datasets Curated Breast Imaging Subset of DDSM (CBIS-DDSM). The first step is to perform preprocessing, which includes image enhancing techniques and the removal of pectoral muscles and labels. The dataset is then annotated, augmented, and divided into 60% for training, 30% for validation, and 10% for testing. The experiment is then performed using a batch size of 8, a learning rate of 0.01, a momentum of 0.843, and an epoch value of 300. To evaluate the performance of our proposed model, our proposed model is compared with YOLOv3 and faster RCNN. The results show that our proposed model performs better than YOLOv3 and faster RCNN with 96% mAP, 93.50% MCC value, 96.50% accuracy, 0.04 FPR, and 0.03 FNR value. The results show that our suggested model successfully identifies and classifies breast tumors while also overcoming previous research limitations by lowering the FPR and FNR and boosting the MCC value.

## 1. Introduction

People nowadays are concerned about their health [1–4]. Today's society faces several challenges related to chronic condition health care issues [5–7]. There is a huge surge see recently in various diseases such as breast cancer, brain tumor, COVID, Dementia, physical inactivity, and lung cancer [8–11]. Machine learning (ML) and deep learning (DL) are being utilized for brain tumor detection, cervical cancer detection, breast cancer detection, COVID detection, thermal sensation detection, and cognitive health assessment of dementia individuals [12–17]. Breast cancer is defined as the uncontrolled growth of cells in a specific area of the body [1, 18]. Breast cancer is the leading cause of cancer mortality among women worldwide. Among all cancers, breast cancer has the most significant incidence and fatality rate, and it is the world's second most common cancer. Every year, around 14.1 million individuals worldwide are diagnosed with breast cancer, with 8.2 million dying as a result. 70% of newly reported cancer cases occur in developing nations, and it is anticipated that by 2025; there will be around 19.3 million newly reported cancer cases yearly [19].

The article "Breast Tumor Detection and Classification in Mammogram Images Using Modified YOLOv5 Network" was retracted in 2023. Reasons: unreliable results or conclusions; concerns about the data; concerns about the peer review; concerns about the citations.

Benign and malignant are two types of breast tumors: benign tumor, in which cancerous cells remain in place and have not extended to surroundings [20]. There is a possibility that that cancerous spread and grow to become malignant. A benign tumor can be easily treated and is not that serious compared to a malignant tumor: a malignant tumor in which cancerous cells spread throughout the body through the circulatory system and cause death. This is the most dangerous type of breast cancer, and most females suffer from this type of tumor. Most breast cancers are malignant.

Breast cancer can be treatable if taken precautions at the proper time. One of the ways of preventing the rapid growth of cells (benign tumor) from becoming full-blown cancer (malignant tumor) and preventing the more spread of cells (malignant tumor) to other organs of the body is early detection. There are effective techniques available to find out the presence of cancer.

Mammography is one of the most commonly used techniques for breast cancer screening which has made a significant contribution to reducing mortality rates through early cancer detection. Mammography [21] is like an X-ray of the breast in which breast compressed between 2 plates and two views of each breast are taken, bilateral craniocaudal (CC) and mediolateral oblique (MLO) [22]. However, the complexity of mammography and the vast amount of tests per radiologist can result in a false diagnosis.

Many researchers have worked hard to create a network that can precisely detect breast tumors with good results, but there is still a significant research gap related to false positive rate, false negative rate, and MCC value. MCC only gives a high score if the prediction performed well in all four categories of the confusion matrix. Because MCC is a more reliable performance metric than accuracy in binary classification, it should be enhanced by decreasing FPR and FNR rates.

The article "Breast Tumor Detection and Classification in Mammogram Images Using Modified YOLOv5 Network" was retracted in 2023. Reasons: unreliable results or conclusions; concerns about the data; concerns about the peer review; concerns about the citations.

The main contributions of this study are as follows:

1. Propose a model that can precisely detect and classify breast tumors into benign and malignant on mammograms
2. Reduce false positive rate (FPR) and false negative rate (FNR) without reducing the degree of accuracy and precision
3. To boost the value of the Matthews correlation coefficient (MCC)
4. Implement all four variants of the YOLOv5 model to determine the most suitable model for detecting and classifying breast tumors
5. Compare our proposed model with state-of-the-art networks to evaluate performance

The rest of the paper is organized as follows: literature review in Section 2.  Section 3 introduces our proposed methodology.  Section 4 provides the outcomes of experimental analysis and results. Finally, conclusions and future work are discussed in Section 5.

## 2. Related Work

In this paper [23], the author suggested a model for the classification of breast masses using the CAD method. MIAS, self-collected datasets, and DDSM datasets are used in this study. Preprocessing, segmentation, collection, and grouping of functions are used in this system. The CAD system includes a CNN model consisting of eight coevolutionary, four max-pooling, and two fully connected layers. The results obtained are then compared to the pretrained nets, Alex Net and VGG16, demonstrating that the proposed CNN achieved higher accuracy and AUC than these two models. The proposed model achieved accuracies of 92.54%, 96.47%, and 95% and AUC scores of 0.85, 0.96, and 0.94 for MIAS, DDSM, and the self-collected dataset, respectively. An extreme learning strategy was used to map the feature fusion and extract the CNN features for breast cancer detection and classification.

In this paper [23], an author has suggested a method to detect breast cancer from mammograms. Preprocessing, segmentation, extraction of features, and classification are used in this research. Next, the image is analyzed, and then the segmentation is added. Second, characteristics are derived, and, thirdly, classification is carried out. Once the findings have been achieved, a distinction is made between various classification methods. Support vector machine (SVM), AdaBoost, decision tree, logistic regression, *K* nearest neighbor, and random forest classifiers are used to classify breast cancer. The accuracy obtained is 90%, 57%, 54%, 85%, 76%, and 61% for support vector machine (SVM), AdaBoost, decision tree, logistic regression, *K* nearest neighbor, and random forest classifiers, respectively, which means that SVM achieves the highest accuracy of all.

The article "Breast Tumor Detection and Classification in Mammogram Images Using Modified YOLOv5 Network" was retracted in 2023. Reasons: unreliable results or conclusions; concerns about the data; concerns about the peer review; concerns about the citations.

In this paper [24], an author proposed a method to classify breast cancer tumors using AGAN for data augmentation and CNN for classification of the tumor. Pattern detection and machine learning techniques such as deep convolutional networks have overtaken state of the art in many visual recognition tasks. This method got 89.17% accurate results but 19.41% false positive rate of classification. In this paper [25], an author proposed a method to detect breast cancer tumors using faster RCNN on OMI-H, OMI-GE, and INbreast datasets. The results achieved using this method are 93% sensitivity for OMI-H, 91% sensitivity for OMI-GE, and 99% sensitivity for INbreast but FPR and FNR rates for OMI-GE dataset increases to 12% and 20%, for INbreast dataset increases to 20% and 29%, and FNR rate for OMI-H increases to 13%, respectively. In this paper [26], an author proposed a method to classify breast cancer tumors using the VGG-16 network on the CBIS-DDSM dataset. This method achieved 82% accuracy, but the drawback is that their MCC value is 63%, FPR is high, 22%, and FNR is 15%.

In this paper [27], an author has suggested a method for identifying breast cancer in mammograms. Noise reduction, segmentation, and grouping are the steps of the proposed model. Gaussian filter is used to eliminate noise from mammogram images. Then, fuzzy *C* means that the clustering algorithm is used for the segmentation of the breast tumor. The Bi-Directional Long-Term Memory Network (Bi-LSTM) classifier is used to diagnose breast cancer with optimized parameters using elephant herding optimization (EHO). MIAS dataset is used in this research. Results are then compared with CNN, DCNN, and Bi-LSTM, from which EHOBi-LSTM got good results, but FPR and FNR rates need to decrease.

In this paper [28], an author proposed a method to detect breast cancer tumors using Dense-Net-169 and Efficient-Net-B5 on a private dataset. This method achieved good accuracy 95.2% for Dense-Net-169 and 95.4% for Efficient-Net-B5, but the drawback is that their FPR and FNR for Dense-Net-169 are high, which is 12% and 13%, respectively. MCC value for both the networks also drops to 66.5% for Dense-Net-169 and 76% for Efficient-Net-B5. In this paper [29], an author suggested a model for identifying, classifying, and segmenting the cancerous area of mammograms. For this study, MIAS and CBIS-DDSM datasets are used. The dataset of images in this research is small. Preprocessing includes the removal of noise, artifacts, and muscle regions that can create a high false-positive rate. A median filter is used to eliminate noise from mammograms. Muscles are separated from the images to clear the tumor, and the images are translated to 512 × 512 patches. To improve system efficiency, the preprocessed image is transformed into 512Ã-512 patches. DL models MASK-RCNN and Deep Lab are then used to identify the tumor. The findings of this study are AUC 0.98 for MASK-RCNN and 0.95 for Deep Lab. The mean average accuracy for the segmentation task is 0.80 and 0.75. The accuracy of the radiologist ranged from 0.80 to 0.88. So, this research is helpful for radiologists in the case of breast tumor classification, but still, results need to improve.

The article "Breast Tumor Detection and Classification in Mammogram Images Using Modified YOLOv5 Network" was retracted in 2023. Reasons: unreliable results or conclusions; concerns about the data; concerns about the peer review; concerns about the citations.

In this paper [30], an author proposed a method to detect breast cancer tumors using a YOLO detector on DDSM and in breast datasets. This method achieved good results that are 99.28% *F*-score for DDSM and 98.02% *F*-score for INbreast dataset, but the drawback is that its FPR is high, which is 14%. A method was also proposed to classify a tumor further using feedforward CNN, ResNet-50, and Inception ResNet-V2. All these three methods got 90+ accuracies for both datasets, but the limitation is that for the breast dataset, FPR increased to 28.57% for CNN, 14.28% for Res-Net50, and 16.66% for Inception ResNet V2. In this paper [2], an author proposed a method to segment and classified breast cancer tumors using Firefly updated chicken-based CSO (FC-CSO) and RCNN on the MIAS dataset. This method achieved good accuracy 93%, sensitivity 97%, specificity 92%, FPR 7%, and FNR 3%, but the drawback is that its MCC value drops to 85%. In this paper [31], an author proposed a method to extract features and classify breast cancer tumors using the CNN model on the MIAS dataset. This method achieved good results: accuracy 95%, sensitivity 98%, specificity 90%, and FNR 2%, but the drawback is that its MCC value drops to 89% and FPR drops to 10%.

In this paper [32], an author proposed a method for the detection of breast cancer tumors using Mobile Net on DDSM and CBIS-DDSM datasets. This method achieved 74.5% accuracy, 76% sensitivity, and 70% precision for CBIS-DDSM dataset and 86.8% accuracy, 95% sensitivity for DDSM dataset but FNR value for CBIS-DDSM dataset increased to 24%.

In this paper [33], an author proposed a method for detection and classification of breast cancer tumors using faster R-CNN and CNN on a private dataset. This method achieved 91.86% accuracy and 94.67% sensitivity. However, the drawback is that their specificity value drops to 89.69%, FPR value increases to 10.3%, and precision value drops to 87.65%. So, results need to improve here. In this paper [34], an author proposed a method for classification of breast cancer tumors using VGG for feature extraction and multiview feature fusion- (MVFF-) based CADx for further classification on MIAS and CBIS-DDSM datasets. The results achieved from this method are accuracy 77.66%, sensitivity 81.82%, and specificity 72.02%. Its FPR and FNR values also increased to 27.9% and 18.18%, respectively. So, the overall result needs to improve here. In this paper [35], an author proposed a method for the classification of breast cancer tumors using CNN on a private dataset. The model achieved sensitivity 91.3% and accuracy 82.4%. Its specificity and MCC value decreased to 56.9% and 51.8%, respectively, and its FPR increased to 43.1%. So, results need to improve here.

The article "Breast Tumor Detection and Classification in Mammogram Images Using Modified YOLOv5 Network" was retracted in 2023. Reasons: unreliable results or conclusions; concerns about the data; concerns about the peer review; concerns about the citations.

In this paper [36], an author proposed a method for segmentation and classification of breast cancer tumors using the multithreshold technique and PNN on MIAS and BCDR datasets. The model achieved sensitivity 98.30%, FNR 1.7%, and accuracy 97.08%. Its specificity decreased to 89.8%, and its FPR increased to 10.2%. So, results need to improve here. In this paper [37], an author proposed a method for the classification of breast cancer tumors using VGG and ResNet-50 on the IRMA dataset. The models achieved accuracies and sensitivities are 94% for VGG-16, 91.7% for ResNet-50% and 99% for VGG-16, and 94% for ResNet-50%, respectively. Its precision for VGG and ResNet-50 decreased to 89% and 88%, respectively. So, results need to improve here. In this paper [38], an author proposed a method for preprocessing and classification of breast cancer tumors using the LBP algorithm and CNN model on the DDSM dataset. The model achieved sensitivity 96.81%, specificity 95.83%, accuracy 96.32%, FPR 4%, and FNR 3%. However, its MCC value drops to 88.48%. So, this is the gap in their research that needs to be improved.

Several researchers have implemented different networks to detect breast tumors and classified them as benign or malignant. Detection and classification accuracies ranging from 90% to 99% were achieved. However, focus on one essential factor is still missing: the false classification ratio and MCC value. In most studies, the false classification ratio is high, and the MCC value is low. Many difficulties arise as a result of fluctuations in these values. If a patient has a benign tumor and the system diagnoses it as a malignant tumor, the patient will be subjected to all of the painful procedures (biopsies, surgeries, and chemotherapies) required to remove the malignant tumor—the same as with a malignant patient. If the machine misidentifies a malignant tumor as benign, the patient will be in danger. This is due to an increase in the false classification ratio and a decrease in the more trustworthy MCC value. As a result, it is essential to build a system that can accurately detect and categorize breast tumors with low FPR and FNR values and high MCC values to more authenticate our research.

The article "Breast Tumor Detection and Classification in Mammogram Images Using Modified YOLOv5 Network" was retracted in 2023. Reasons: unreliable results or conclusions; concerns about the data; concerns about the peer review; concerns about the citations.

## 3. Proposed Methodology

The primary goal of this study is to create a model that can effectively detect and classify breast tumors while also minimizing FPR and FNR rates and increasing MCC values. The CBIS-DDSM [26] dataset is utilized for this. As seen in Figure 1, the initial stage is to remove the rough white borders, followed by the removal of artifacts and pectoral muscles. CLAHE is useful for image enhancement. The images are then subjected to erosion, a morphological procedure. Annotation is completed with augmentation after images have been cleaned and enhanced. The prepared data is then fed into our proposed YOLOv5 model. In this study, all four versions of YOLOv5 are utilized. The original version of YOLOv5 is then compared to modified variants of YOLOv5. After a comparison of the original and modified versions, a comparison with a state-of-the-art network is performed.

### 3.1. Dataset Description

The Curated Breast Imaging Subset of DDSM (CBIS-DDSM) dataset comprises 10239 images, including whole mammograms, cropped images, and ROI mask images with mass and calcification are utilized in this study. This study utilized 2424 complete mammograms of benign and malignant masses (as showing in Figure 2 to implement our proposed model, leaving microcalcification for future research). Data augmentation is a technique used in image processing to produce extra training data from current data. Augmentation is done in this study by flipping pictures horizontally, rotating them at 90 and 180 degrees, and making various copies. A total of 4865 pictures were created after augmentation. 60% of data is used for training, 30% is used for validation, and 10% is used for testing. Because of the Graphics Processing Unit, we chose to build our model, which cannot handle huge pictures, and the size of the images has been decreased from 3000 × 4500 pixels to 1000 × 2000 pixels.

### 3.2. Preprocessing

Before implementing our proposed model, preprocessing is performed with the following few steps.

#### 3.2.1. Removal of White Borders

To begin, images are thoroughly cleaned using several approaches. Images have a rough outside border with white lines, indicated with red lines, as shown in Figure 3. Because the white color in mammograms also represents tumors, it can lead to misdiagnosis of benign and malignant tumors.

White lines are eliminated to avoid misclassification by cropping the image area somewhat using the cropping function. Images are shown in Figure 4 after removing harsh white lines.

The article "Breast Tumor Detection and Classification in Mammogram Images Using Modified YOLOv5 Network" was retracted in 2023. Reasons: unreliable results or conclusions; concerns about the data; concerns about the peer review; concerns about the citations.

#### 3.2.2. Removal of Artifacts and Pectoral Muscles

Because pectoral muscles and artifacts have the same intensity as the tumor region, removing them from mammograms is the most challenging task [39]. To locate the actual tumor area, pectoral muscles and artifacts must be removed. After cropping white lines, artifacts and pectoral muscles are removed using intensity value on specific columns in mammograms as shown in Figure 5.In Matrix Laboratory (MATLAB), the left pectoral muscles and labels are removed individually, as are the right pectoral muscles and labels.

#### 3.2.3. Contrast Limited Adaptive Histogram Equalization (CLAHE)

After the pectoral muscles and labels have been removed, Contrast Limited Adaptive Histogram Equalization (CLAHE) [40] is utilized to improve the mammography. Image enhancement plays an essential role in medical imaging since it allows us to see hidden features in an image. So, in this study, CLAHE is utilized to enhance mammograms and provides the best results in viewing the tumor part. CLAHE works using tiles, which are small sections of a larger image rather than the entire image. The adjacent tiles are blended using bilinear interpolation to remove the false boundaries. When utilizing CLAHE, there are two factors to keep in mind. The first is clip limit, which sets the contrast threshold value to 40 by default. The second one is tile grid size, which sets the number of tiles in the row and column, and 8 × 8 is its default value.  Figure 6 shows an image before and after applying CLAHE.

#### 3.2.4. Morphological Operation

Morphological image processing [41] is a set of nonlinear procedures that deal with the structure or morphology of image features. Morphological operations are often used to remove minor features from a picture while retaining more extensive details. There are a variety of morphological operations. In this study, morphological operations are required to remove surrounding tissues to make the tumor part apparent; so, erosion is utilized in this research to make the tumor part prominent while removing the unnecessary tiny tissue elements.  Figure 7 shows an image before and after applying morphological erosion operation.

(1) $$\begin{array}{c} X!Y=\left\{c\in W\;|\;Y_{c}\subseteq X\right\}. \end{array}$$

Equation (1) shows erosion of binary image *X* by the structuring element *Y*. *W* is a Euclidean space, and *X* is a binary image in *W* where *Y*_*c* is the translation of *Y* by the vector *c* showing in equation (2).

(2) $$\begin{array}{c} Y_{c}=\left\{y+c\;|\;y\in Y\right\},\forall c\in W. \end{array}$$

### 3.3. Annotation

After morphological operations, the dataset is prepared for use in tumor detection and classification. The Yolov5 model is utilized in this study to detect and classify breast tumors, and we need annotated data to utilize this model. As a result, data is being annotated utilizing an online source called Roboflow. Square boxes are used to annotate images. The annotated data is shown in Figure 8. Annotated data has two types of files. One is an image file, and the second one is a text (.txt) file. The text file contains the dimensions of the square on a tumor. The sample is shown in Figure 9.

The article "Breast Tumor Detection and Classification in Mammogram Images Using Modified YOLOv5 Network" was retracted in 2023. Reasons: unreliable results or conclusions; concerns about the data; concerns about the peer review; concerns about the citations.

### 3.4. YOLOv5

The YOLO neural network design predicts a collection of bounding boxes and class probabilities. First, it splits the entire image into many grids of varying sizes, and anchor boxes are produced in each grid of the input image using a predefined scale and size. Compared to a two-stage detector, each anchor box predicts the objectness score and box center offset *x*, box center offset *y*, box width, box height, and class scores all at once. Thus, YOLO is a one-stage object detector that is a rapid end-to-end technique for detecting objects. There are many versions of YOLO. In this paper, YOLOv5 is used for the detection and classification of breast tumors. The YOLOv5 architecture contains four architectures, specifically named YOLOv5s, YOLOv5m, YOLOv5l, and YOLOv5x, respectively. The main difference among them is that the amount of feature extraction modules and convolution kernel in the specific location of the network is different. The size of models and the number of model parameters in the four architectures increase in turn as showing in Table 1. The basic structure of YOLOv5 (YOLOv5s) is shown in Figure 10.

In this research, all 4 versions of YOLOv5 are used for the detection and classification of breast tumors and to make a comparison between these 4 versions. Let us start with yolov5s.

(3) $$\begin{array}{c} A=\mathrm{Min}\left(\frac{C_{1}}{C_{0}},\frac{B_{1}}{B_{0}}\right), \end{array}$$

(4) $$\begin{array}{c} R=\text{np}.\mathrm{mod}\left(\frac{C_{1}}{A},\frac{B_{1}}{A}\right), \end{array}$$

(5) $$\begin{array}{c} C_{1}\times \left(B_{1}+R\right). \end{array}$$

Equations (3)–(5) are showing the method of mosaic data enhancement. *C*_0 and *B*_0 is the original image size. *C*_1 and *B*_1 are the original image scale size, *A* is the scale factor, and *R* is the gray filled value.

It has three important parts like any other single-stage object detector as showing in Figure 10.

- Model backbone
- Model neck
- Model head

Model backbone is mainly used to extract key features from an input image. The focusing layer is the initial layer of the backbone network, and it is used to simplify the model calculation and boost training speed. It serves the following purposes: using a slicing technique, the three-channel image is first split into four slices of 3 × 320 × 320 each. Second, concatenation is used to connect the four sections indepth, with the output feature map having a size of 12 × 320 × 320, and then the output feature map with a size of 32 × 320 × 320 was formed via the convolutional layer made of 32 convolution kernels. Finally, the findings are output into the next layer via the BN layer (batch normalization) and the Hardswish activation functions. The BottleneckCSP [42] module is the third layer of the backbone network, and it is designed to extract the image's indepth information more effectively. The BottleneckCSP module is primarily formed of a Bottleneck module, as shown in Figure 11, which is a residual network architecture that joins a convolutional layer (Conv2d + BN + ReLu activation function) with a convolution kernel size of 1 × 1 with a convolution kernel size of 3 × 3. The final output of the Bottleneck module is the sum of this part's output and the initial input via the residual structure.

(6) $$\begin{array}{c} A_{1}=B_{1}\times A_{0}, \end{array}$$

(7) $$\begin{array}{c} A_{2}=B_{2}\times \left[A_{0},A_{1}\right], \end{array}$$

(8) $$\begin{array}{c} A_{k}=B_{k}\times \left[A_{0},A_{1},\cdots ,A_{k}-1\right]. \end{array}$$

Equations (6)–(8) are showing the working of CSP network from 1st layer to the last layer. Asterisk sign shows the operator, and [*A*_0, *A*_1, ⋯] means concatenating [*A*_0, *A*_1, ⋯], and *B*_i and *A*_*i* are the weights and output of the *i*-th dense layer, respectively. The first input of the BottleneckCSP module is split into two branches, and the number of feature map channels is halved using convolution in two branches as shown in Figure 12. The output feature map of branches one and two is then connected in depth using concat through the Bottleneck module and Conv2d layer inbranch two. Finally, the module's output feature map is created after progressively passing through the BN layer and Conv2d layer, and the size of this feature map is the same as the size of the BottleneckCSP module's input.

The article "Breast Tumor Detection and Classification in Mammogram Images Using Modified YOLOv5 Network" was retracted in 2023. Reasons: unreliable results or conclusions; concerns about the data; concerns about the peer review; concerns about the citations.

The SPP module (spatial pyramid pooling) [43] is the ninth layer of the Backbone network, and it is designed to increase the network's receptive field by transforming any size of the feature map into a fixed-size feature vector. Following a cycle through the convolutional layer, the feature map with a size of 256 × 20 × 20 is output; the convolution kernel size is 1 × 1. Then, this feature map and the output feature map are connected indepth after being subsampled through three concurrent maxpooling layers, and the size of the output feature map is 1024 × 20 × 20.

The model neck is mainly used to create feature pyramids. Feature pyramids assist models in successfully generalizing when it comes to object scaling, and it facilitates the identification of the same object in various sizes and scales.

(9) $$\begin{array}{c} A=A_{0}+\text{lo}{\text{g}}_{2}\left(\frac{\sqrt{x}y}{224}\right). \end{array}$$

Equation (9) is used to select the feature map. Feature pyramids are pretty beneficial in assisting models to perform well on unknown data. The model head is primarily responsible for the final detection step, and it uses anchor boxes to construct final output vectors with class probabilities, objectness scores, and bounding boxes. The detection network of the YOLOv5s structure comprises three detect layers, each with an input of a feature map with dimensions of 80 × 80, 40 × 40, and 20 × 20 utilized to detect image objects of various sizes. Each detects layer outputs a 21-channel vector with two classes, 1 class probability, four surrounding box position coordinates, and three anchor boxes. Then, the predicted bounding boxes and categories of the targets in the original image were generated and labeled, allowing the detection of the images' targets to be implemented.

### 3.5. Improvement in the YOLOv5 Model

The YOLOv5 Model does not produce the desired results in its original form. Even on complex surfaces, the model should detect and categorize tumors correctly. The model's size must also be reduced as much as possible in order for it to be deployed in hardware devices. As a result, we make some changes to the model's backbone. The YOLOv5s architecture's backbone network comprises four BottleneckCSP modules, each with numerous convolutional layers. Although the convolution procedure can extract image features, the convolution kernel has many parameters, resulting in many parameters in the recognition model. As a result, the convolutional layer on the original CSP module's different branch is deleted. The BottleneckCSP module's input feature map is directly connected with the output feature map with another branch indepth, significantly reducing the number of parameters in the module. The architecture of the improved BottleneckCSP module is shown in Figure 13.

In the study, four stages of the original backbone network where the BottleneckCSP module is used are replaced with four BottleneckCSP-new modules, as shown in Figure 14, to justify the limitation of BottleneckCSP-new, which may end up causing deficiency in the extraction of deep features in the image due to its lightweight attributes.

(10) $$\begin{array}{c} \text{Con}.=P\left(\text{Tumor}\right)\times \text{Los}{\text{s}}_{p}. \end{array}$$

Equation (10) shows the function of calculation of loss. Con. denotes confidence, while *P* (Tumor) denotes the likelihood that the grid cell has a tumor. When the model is trained, the value is one if the target's center lies in a grid cell. Otherwise, it is 0. The loss value computes the change between the anticipated bounding box and the grid cell's ground truth box.

(11) $$\begin{array}{c} \text{IoU}=\frac{A\cap B}{A\cup B}, \end{array}$$

(12) $$\begin{array}{c} L_{\text{GIOU}}=1-\text{IoU}+\frac{\left|A-B\cup B^{f}\right|}{\;|\;X\;|\;}. \end{array}$$

IoU is the junction and unity of two boxes, and this is a standard statistic for describing the degree of coincidence between two boxes. The calculation method is shown in equation (11). GIoU loss function is used in this study, and the calculation method is shown in equation (12).

The article "Breast Tumor Detection and Classification in Mammogram Images Using Modified YOLOv5 Network" was retracted in 2023. Reasons: unreliable results or conclusions; concerns about the data; concerns about the peer review; concerns about the citations.

## 4. Experimental Analysis and Results

In our experiment, we begin by annotating data. Annotating the data involves highlighting a particular object (tumor) on the dataset's images. We split the data into three sections. 60% of the data is used for training, 30% for validation, and 10% for testing. In YOLOv5, there are four models: YOLOv5s, YOLOv5m, YOLOv5l, and YOLOv5x. The upgraded version of the YOLOv5 model is trained on Nvidia GPU using PyCharm frame 2020 of version 1.4.0 and Python 3.6 to train and test the breast tumor detection and classification model as calling CUDA, Cudnn, OpenCV, and other needed libraries. The experimental setup is Linux Ubuntu 16.04, with a GeForce GTX 1080Ti 11GB graphics card. The software used the Windows 10 operating system, the Keras deep learning framework, and the TensorFlow deep learning framework. The YOLOv5 model, a pretrained checkpoint on the COCO dataset, was fine-tuned. Stochastic Gradient Descent [44] is the optimizer utilized for this model (SGD). The model training batch size is set to 8, the learning rate is set to 0.01, the momentum is set to 0.843, and the decay rate is set to 0.00036. The IOU (intersection over union) value is set at 0.2. The training epoch value is set to 300. The model is trained consistently and performed well. After training, the weight file for this model is saved, and the test set is used to evaluate the model's performance. The network's final output is the position boxes of the two types of breast tumors (benign and malignant), as well as the likelihood of belonging to a given category.

### 4.1. Performance Measure

Different measures are used to evaluate the performance of the model. Accuracy [45], mAP, sensitivity 13, specificity, *F*-measure [46], MCC [47] measurements are taken using TP (true positive), TN (true negative), FP (false positive), and FN (false negative).

The article "Breast Tumor Detection and Classification in Mammogram Images Using Modified YOLOv5 Network" was retracted in 2023. Reasons: unreliable results or conclusions; concerns about the data; concerns about the peer review; concerns about the citations.

TP (true positive): the number of cases accurately defined in this section.

TN (true negative): the number of examples correctly refused in this section.

FP (false positive): the number of cases unfairly denied in that class.

FN (false negative): the number of instances wrongly listed in that class.

FPR (false positive rate): the results say you have the disease, but you do not.

FNR (false negative rate): the results say you do not have a disease, but you really do.

(13) $$\begin{array}{c} \text{Sensitivity}=\frac{\text{TP}}{\text{TP}+\text{FN}}, \end{array}$$

(14) $$\begin{array}{c} \text{Specificity}=\frac{\text{TN}}{\text{FP}+\text{TN}}, \end{array}$$

(15) $$\begin{array}{c} \text{Precision}=\frac{\text{TP}}{\text{FP}+\text{TP}}, \end{array}$$

(16) $$\begin{array}{c} m\text{AP}=\frac{1}{N}\overset{N}{\underset{i=1}{\sum }}\text{A}{\text{P}}_{i}, \end{array}$$

(17) $$\begin{array}{c} \text{Accuracy}=\frac{\text{TN}+\text{TP}}{\text{FP}+\text{TN}+\text{FN}+\text{TP}}, \end{array}$$

(18) $$\begin{array}{c} F-measure=\frac{2\left(Sensitivity\right)\left(Precision\right)}{Sensitivity+Precision}, \end{array}$$

(19) $$\begin{array}{c} \text{MCC}=\frac{\left(\text{TP}\right)\left(\text{TN}\right)-\left(\text{FP}\right)\left(\text{FN}\right)}{\sqrt{\left(\text{TP}+\text{FP}\right)\left(\text{TP}+\text{FN}\right)\left(\text{TN}+\text{FP}\right)\left(\text{TN}+\text{FN}\right)},} \end{array}$$

(20) $$\begin{array}{c} \text{FPR}=1-\text{Specificity}=\frac{\text{FP}}{\text{FP}+\text{TN}}, \end{array}$$

(21) $$\begin{array}{c} \text{FNR}=1-\text{Sensitivity}=\frac{\text{FN}}{\text{TP}+\text{FN}}. \end{array}$$

Equations (13)–(21), represent sensitivity, specificity, precision, mAP, accuracy, *F*-measure, MCC, FPR, and FNR, respectively.

MCC value is the primary and most essential performance metric. Instead, the Matthews correlation coefficient (MCC) is a more reliable statistical rate in binary classification that yields a high score only if the prediction performed well in all four confusion matrix categories.

The mAP is an essential parameter for measuring network model training, and it is the average mean precision of each AP category. AP denotes the region contained by precision and recall as two-axis mapping, the average is denoted by *M*, and the number after @ is the threshold for evaluating IoU as positive and negative samples.

### 4.2. Comparison of Original YOLOv5s and Modified YOLOv5s

Modified YOLOv5s performs better than original YOLOv5s. As seen in Figure 15, modified YOLOv5s achieve 95% sensitivity, 97% specificity, 96.93% precision, 95.20% mAP, 96% accuracy, and 92.02% MCC value. Original YOLOv5s achieve 90% sensitivity, 91% specificity, 90.90% precision, 88.70% mAP, 90.50% accuracy, and 81% MCC value.

The article "Breast Tumor Detection and Classification in Mammogram Images Using Modified YOLOv5 Network" was retracted in 2023. Reasons: unreliable results or conclusions; concerns about the data; concerns about the peer review; concerns about the citations.

### 4.3. Comparison of Original YOLOv5m and Modified YOLOv5m

As seen in Figure 16, modified YOLOv5m achieves 94% sensitivity, 97% specificity, 96.90% precision, 95% mAP, 95.50% accuracy, and 91.04% MCC value. Original YOLOv5m achieves 91% sensitivity, 89% specificity, 89.21% precision, 87.20% mAP, 90% accuracy, and 80.02% MCC value. Modified YOLOv5m performs well as compared to original YOLOv5m.

### 4.4. Comparison of Original YOLOv5l and Modified YOLOv5l

As seen in Figure 17, modified YOLOv5l achieves 95% sensitivity, 97% secificity, 96.93% precision, 95.20% mAP, 96% accuracy, and 92.02% MCC value. Original YOLOv5l achieves 92% sensitivity, 91% specificity, 91.08% precision, 88.90% mAP, 91.5% accuracy, and 83% MCC value. Modified YOLOv5l performs well as compared to the original YOLOv5l.

### 4.5. Comparison of Original YOLOv5x and Modified YOLOv5x

As seen in Figure 18, modified YOLOv5x achieves 96% sensitivity, 97% specificity, 97% precision, 96% mAP, 96.50% accuracy, and 93.60% MCC value. Original YOLOv5x achieves 93% sensitivity, 92% specificity, 92.07% precision, 89.20% mAP, 92.5% accuracy, and 85% MCC value. Modified YOLOv5x performs well as compared to original YOLOv5x.

The next performance measure is FPR and FNR rates, and these two rates should be low to authenticate our results. Here in this study, FPR and FNR rates for all four versions of modified YOLOv5 and original YOLOv5 are mentioned in Table 2.

### 4.6. Comparison of Modified YOLOv5x, YOLOv3, and Faster RCNN

We use three detection models for breast tumor detection and compare their performance: YOLOv5, faster R-CNN, and Yolov3. First, we compared all variants of the original YOLOv5 and modified YOLOv5. Then, we compare all four versions of modified YOLOv5, and we find that modified YOLOv5x outperformed all other versions. As a result, for further comparisons with faster RCNN and YoloV3, we utilize modified YOLOvx.  Table 3 shows that modified YOLOv5x has the lowest FPR and FNR rates than YOLOv3 and faster RCNN. MCC, accuracy, and mAP that we achieve for modified YOLOv5x are 93.50%, 96.50%, and 96%, respectively, higher than the other two detection models. So, it is clear that modified YOLOvx performs better than faster RCNN and YOLOv3 to detect and classify breast tumors.

The YOLOv5 model detects and categorizes breast tumors into two classes. There are two types of tumors: benign and malignant. All four YOLOv5 variants are used to detect and classify breast tumors. The results obtained are not satisfactory, which is why all four versions of YOLOv5 have been updated. It is discovered that modified versions outperform the originals, and YOLOv5x performs well among modified versions compared to other modified versions.  Figure 19 depicts the results of breast tumor detection and classification using an enhanced YOLOv5x network.

The article "Breast Tumor Detection and Classification in Mammogram Images Using Modified YOLOv5 Network" was retracted in 2023. Reasons: unreliable results or conclusions; concerns about the data; concerns about the peer review; concerns about the citations.

## 5. Conclusion

Early detection and classification of breast tumors are increasingly required to reduce the risk of death among cancer patients. Many researchers have conducted extensive research and proposed models for detecting and classifying benign and malignant breast tumors, but something is still missing. In many studies, the model reached a performance accuracy of 90% or higher, but even though the MCC value decreased, the FPR and FNR were increased. Rates of FPR and FNR should be as low as possible. Because the MCC value is a more accurate measure for binary classification than accuracy, it should be enhanced to validate our findings further. This paper proposes a lightweight detection and classification method based on improved YOLOv5 to detect and classify breast tumors. All four versions (YOLOv5s, YOLOv5m, YOLOv5l, YOLOv5x) of modified YOLOv5 are used in this study. BottleneckCSP module is updated to BottleneckCSP-new module, which is utilized to replace the BottleneckCSP module in the backbone architecture of the original YOLOv5s network to improve results and make the network lighter. To evaluate performance, the original YOLOv5 and the modified YOLOv5 are compared.

The results show that modified versions of YOLOv5 perform better than original YOLOv5. Modified YOLOv5s, YOLOv5m, YOLOv5l, and YOLOv5x achieve (92.02%, 91.04%, 92.02%, 93.60%) MCC value, (0.05, 0.06, 0.05, 0.04) FPR value, and (0.03, 0.03, 0.03, 0.03) FNR value better than the original YOLOv5 model. Among all four modified YOLOv5 versions, YOLOv5x outperforms the other three. So, modified YOLOv5x is compared to faster RCNN and YOLOv3. It has been observed that modified YOLOv5x outperforms faster RCNN and YOLOv3 with 0.04 FPR, 0.03 FNR, 93.60% MCC, 96.50% accuracy, 96% mAP, 97% precision, 96% sensitivity, and 97% specificity. The results conclude that our suggested model successfully identifies and classifies breast tumors while also overcoming previous research limitations by lowering the false positive and false negative ratio and boosting the MCC value.

### 5.1. Future Work

In this work, a modified YOLOv5 model is used to detect and classify breast tumors as benign or malignant, with promising results. Our suggested model can detect tumors that are in shape or those that are lightly shaped. However, our proposed model cannot detect poorly shaped tumors in abnormal images, which is a limitation. We will improve this network in the future to recognize all shapes and sizes of tumors, making it more convenient. We have also just focused on breast mass abnormalities so far. So, the study can be expanded in the future to cover macro calcification anomalies that are not currently evaluated.

The article "Breast Tumor Detection and Classification in Mammogram Images Using Modified YOLOv5 Network" was retracted in 2023. Reasons: unreliable results or conclusions; concerns about the data; concerns about the peer review; concerns about the citations.

## Figures and Tables

**Figure 1:** Proposed flow.

**Figure 2:** Benign and malignant images from CBIS-DDSM dataset.

**Figure 3:** Rough images with white lines.

**Figure 4:** Images after removing white lines.

**Figure 5:** Images with pectoral muscles and labels are on left side and images with removal of pectoral muscles and labels are on the right side.

**Figure 6:** Before and after applying CLAHE, respectively.

**Figure 7:** Before and after applying erosion morphological operation, respectively.

**Figure 8:** Annotated images.

**Figure 9:** Text file details.

**Figure 10:** Architecture of original Yolov5s.

**Figure 11:** Bottleneck module.

**Figure 12:** BottleneckCSP module.

**Figure 13:** Improved BottleneckCSP module.

**Figure 14:** Modified version of YOLOv5.

**Figure 15:** Comparison of modified YOLOv5s with original YOLOv5s on the basis of sensitivity, specificity, accuracy, mAP, precision, and MCC.

**Figure 16:** Comparison of modified YOLOv5m with original YOLOv5m on the basis of sensitivity, specificity, accuracy, mAP, precision, and MCC.

**Figure 17:** Comparison of modified YOLOv5l with original YOLOv5l on the basis of sensitivity, specificity, accuracy, mAP, precision, and MCC.

**Figure 18:** Comparison of modified YOLOv5x with original YOLOv5x on the basis of sensitivity, specificity, accuracy, mAP, precision, and MCC.

**Figure 19:** Results of breast tumor detection and classification using improved YOLOv5x network.

**Table 1:** Difference between four versions of YOLOv5.

	YOLOv5s	YOLOv5m	YOLOv5l	YOLOv5x
CSP1	CSP1-1	CSP1-2	CSP1-3	CSP1-4
CSP1	CSP1-3	CSP1-6	CSP1-9	CSP1-12
CSP1	CSP1-3	CSP1-6	CSP1-9	CSP1-12
CSP2	CSP2-1	CSP2-2	CSP2-3	CSP2-4
CSP2	CSP2-1	CSP2-2	CSP2-3	CSP2-4
CSP2	CSP2-1	CSP2-2	CSP2-3	CSP2-4
CSP2	CSP2-1	CSP2-2	CSP2-3	CSP2-4
CSP2	CSP2-1	CSP2-2	CSP2-3	CSP2-4

**Table 2:** Comparison of all four versions of modified YOLOv5 with original YOLOv5 on the basis of false positive rate (FPR) and false negative rate (FNR).

Models	FPR	FNR
Original YOLOv5s	0.09	0.10
Modified YOLOv5s	0.05	0.03
Original YOLOv5m	0.11	0.09
Modified YOLOv5m	0.06	0.03
Original YOLOv5l	0.09	0.08
Modified YOLOv5l	0.05	0.03
Original YOLOv5x	0.08	0.07
Modified YOLOv5x	0.04	0.03

**Table 3:** Comparison of all four versions of modified YOLOv5 with original YOLOv5 on the basis of false positive rate (FPR) and false negative rate (FNR).

Models	FPR	FNR	mAP	MCC	Acc.
Modified YOLOv5x	0.04	0.03	96%	93.50%	96.50%
YOLOv3	0.15	0.19	85%	82.5%	86%
Faster RCNN	0.20	0.15	84.2%	81.7%	85.3%

The article "Breast Tumor Detection and Classification in Mammogram Images Using Modified YOLOv5 Network" was retracted in 2023. Reasons: unreliable results or conclusions; concerns about the data; concerns about the peer review; concerns about the citations.

## Data Availability

The dataset used to support the findings of this study are included within the article.
